The article "Cardioprotection by Citrus grandis (L.) Peel Ethanolic Extract in Alloxan-Induced Cardiotoxicity in Diabetic Rats" was published in 2022. Journal: Biomed Res Int.

# Cardioprotection by Citrus grandis (L.) Peel Ethanolic Extract in Alloxan-Induced Cardiotoxicity in Diabetic Rats

**DOI:** 10.1155/2022/2807337

**Published:** 2022-06-16

**Authors:** Imtiyaz Ahmed Najar, Moomin Hussain Bhat, Zulfqar Lateif Qadrie, Maria John Newton Amaldoss, Ajay Singh Kushwah, Thakur Gurjeet Singh, Atul Kabra, Nadeem Khan, Manish Kumar

**Affiliations:** ^1^Department of Pharmacology, Lovely Professional University, Jalandhar, Punjab 144411, India; ^2^Department of Pharmacology, Swift School of Pharmacy, Rajpura, Punjab 140401, India; ^3^Department of Endocrinology, Sher-I-Kashmir Institute of Medical Sciences (SKIMS) (A Deemed University), Soura, Srinagar, Jammu and Kashmir 190011, India; ^4^Department of Clinical Pharmacology, Sher-I-Kashmir Institute of Medical Sciences (SKIMS) (A Deemed University), Soura, Srinagar, Jammu and Kashmir 190011, India; ^5^Lowy Cancer Research Centre, Prince of Wales Clinical School, University of New South Wales, Sydney, NSW 2052, Australia; ^6^Department of Pharmacology, Amar Shaheed Baba Ajit Singh Jujhar Singh Memorial College of Pharmacy, Bela, Ropar 140111, India; ^7^Chitkara College of Pharmacy, Chitkara University, Punjab 140401, India; ^8^University Institute of Pharma Sciences, Chandigarh University, 140413 Gharuan, Mohali, India

## Abstract

Diabetic cardiomyopathy (DCM) pathogenesis is multifarious, and there are insufficient therapeutic options to treat DCM. The present research explored the effects of Citrus grandis peel ethanolic extract (CGPE) in alloxan-induced DCM in rats. Diabetes was triggered by intraperitoneal (i.p.) injection of alloxan (150 mg/kg) in Wistar rats (200-250 g). CGPE (100, 200, and 400 mg/kg) or glibenclamide (Glib, 10 mg/kg) were administered orally for 2 weeks. After the treatment schedule, prooxidants (thiobarbituric acid reactive substances), antioxidants (glutathione, catalase, and superoxide dismutase), and inflammatory markers (tumor necrosis factor-*α*) were determined in cardiac tissues. Biomarkers of cell death, viz., lactate dehydrogenase (LDH), creatine kinase MB (CK-MB) activity, glucose levels, total cholesterol (TC), and high-density lipoproteins (HDL), were assessed in the blood. Rats administered with alloxan showed a consistent increase in blood glucose level (days 7 and 14) that was lowered considerably (*p* < 0.001) by CGPE or Glib. Alloxan-induced increase in LDH, CK-MB, TC, and decline in HDL was attenuated (*p* < 0.001) in rats that were treated with CGPE or Glib. Alloxan significantly (*p* < 0.001) elevated oxidative stress, inflammation, and reduced antioxidants in the cardiac tissue of rats, and these pathogenic abnormalities were ameliorated (*p* < 0.001) by CGPE. Histopathological studies showed a decrease in morphological disruptions by alloxan in CGPE-treated rats. CGPE (400 mg/kg) significantly ameliorated biochemical parameters in comparison to the lower doses against alloxan cardiotoxicity. Citrus grandis peel extract can be an alternative in the management of DCM.

## 1. Introduction

At an early point, diabetic cardiomyopathy (DCM) is primarily described by myocardial fibrosis and abnormal remodeling, is linked as diastolic dysfunction and then systolic dysfunction, and results in the progression of acute heart failure [1]. DCM is the major cause of diabetes-induced mortality. While the number of diabetes cases continues to grow, new approaches to defend against DCM, which are marked by cardiac hypertrophy, accelerated apoptosis, fibrosis, and impaired insulin metabolism, are desperately required [2]. DCM's exact pathogenesis is complicated and multifaceted. However, early causes contributing to diabetic heart cell mutilation are known to be a consequence of different triggers, i.e., persistently increased blood sugar level, reactive oxygen species (ROS), reactive nitrogen species (RNS), extracellular matrix protein upregulation, myocardium fibrosis, protein kinase C instigation, cytokines, and renin-angiotensin system activation [3]. An imbalance between endogenous ROS as well as the antioxidant system has been reported to contribute to the advancement or progression of DCM [4]. Too much ROS generation, i.e., superoxides can contribute to cardiovascular system (CVS) problems [5]. Because the usage of synthetic medicines to treat this disease and its consequences involves tremendous costs for developing nations' economies with unintended side effects, new approaches are desperately needed. It was also concluded by a study that a diet rich in fruits, vegetables, and spices lowers the risk of cardiovascular death [6].

Another study concluded that proinflammatory cytokines are released in conditions that are associated with myocardial inflammation, such as myocardial ischemia, myocarditis, and idiopathic cardiomyopathies. These cytokines are found to be strong inducers of nitric oxide (NO) synthesis in cardiac myocytes. An increased level of NO has been found to be combined with cell death [7]. It has been reported that the advancement of DCM involves disparities between endogenous ROS as well as the antioxidant system [4].

Novel medications for diabetes management that may link the development of hyperglycemia and diabetic disorder are on the lookout. The World Health Organization (WHO) diabetes expert committee has suggested investigating traditional diabetes management treatments and their complication. In Western countries, too, the use of herbal products is booming, as these are known to be safer [8]. Another consideration is that it is time-intensive and extraordinarily costly to identify new chemical entities. WHO reports that 80 percent of Asian and African communities are already utilizing herbal medicines for their health care needs. Around 28 percent of new chemical entities were found to be natural products or their derivatives between 1987 and 2002 [9]. Recent research findings revealed that dieting loaded with fruits, vegetables, and also spice reduces the cardiovascular risk of death [6]. In the discovery of new medicinal agents from plants, phytochemical research based on ethnopharmacological information is generally considered a sound approach [9].

Research findings had shown that several edible plants (e.g., Embelia ribes and Rooibos) [10], phytoproducts (e.g., green tea), and phytoconstituents (e.g., taxifolin and aspalathin) [11, 12] attenuate cardiac dysfunction [13]. Citrus fruits are often identified for their economic value and pharmaceutical properties. The title Citrus is the common floral genus of Rutaceae owing to the tropical and subtropical kinds of Southeast Asia. The most versatile citrus fruits are mandarins (C. reticulate Blanco), pomelos (C. grandis Osbeck), sour oranges (C. aurantium L.), sweet orange (C. sinensis Osbeck), lime (C. aurantifolia Christm), and lemon (C. limon L.). Citrus fruits are famed for their scent, owing in part to flavonoids and limonoids (which in effect are terpenes) found in the peel, and are recognized as being abundant in many phytonutrients that are important to wellbeing endorsement and illness deterrence [14]. Several investigators conclude that the citrus florae exhibit an array of flavonoid components which are the plants' secondary chemical metabolites. Whilst a wide range of bio-like activities existed for some flavonoids, their protective role in living structures was mainly an outcome of their antioxidant potentials owing to transferring ROS, metal catalyst chelation, antioxidants, and colon cancer [15, 16].

Citrus grandis peel extracts have the properties to be a possible therapeutic mediator for the management of DCM owing to their flavonoids, hypoglycemic function, antioxidant activity, and antiapoptosis mechanisms [17]. In the current experiments, the potency of ethanol extract from Citrus grandis peel in alloxan-induced DCM in rats was explored.

## 2. Methods

### 2.1. Drugs and Chemicals

Glibenclamide (Glib) was procured from Ind-Swift Pvt. Ltd. (India). Alloxan and sodium carboxymethyl cellulose (CMC) were procured from SD Fine Chem Ltd. (SDFCL), Mumbai. Dibasic sodium phosphate, monobasic sodium phosphate, and diethyl ether (A.B. Enterprises, Mumbai); formalin, Folin-Ciocalteu reagent, thiobarbituric acid (TBA), glutathione (GSH), and dimethylsulfoxide (DMSO) (Hi-Media Lab Pvt. Ltd., Mumbai); ethylenediaminetetraacetic acid (EDTA) (Loba Chemie Pvt. Ltd; Mumbai); ethanol (Indian Chemical Co., Delhi); and aluminium trichloride (AlCl_3_), sodium cyanide, sodium hydroxide (NaOH), sodium nitroprusside, sodium nitrite (NaNO_2_), and sodium carbonate (Na_2_CO_3_) (Sisco Research Laboratory, Mumbai) were procured. Total cholesterol kit, HDL kit, and total protein kit were procured from Avecon Healthcare Pvt. Ltd., Saha (Ambala). The lactate dehydrogenase kit was procured from Reckon Diagnostics Pvt. Ltd., Gorwa, Vadodara. Creatine kinase isoenzyme (CKMB) was procured from Coral Clinical Systems, Industrial Estate, Verna, Goa.

### 2.2. Investigational Animals

Male Wistar rats (200-250 g; age 5-6 months) were acquired from the National Institute of Pharmaceutical Education and Science, Mohali (Punjab). All the animals were quarantined and their health was monitored for one week. The rats were housed under standard laboratory conditions at the institute's Central Animal Facility (CAF), viz., temperature, 23 ± 2°C; humidity, 40 ± 10%; and artificial light-dark period, 12 hours each (8 : 00 AM to 8 : 00 PM). The Institutional Animal Ethics Committee (SSP/IAEC/17/02) authorized the investigational procedure of this research, and experiments were conducted as per the guiding principles of the Committee for the Purpose of Control and Supervision of Experiments on Animals (CPCSEA), Ministry of Forests and Climate, Government of India, and Indian National Science Academy. All the animals were given an acclimatization period of 14 days before the initiation of the experiments. According to the guidelines of CPCSEA, animals were nourished with a normal rodent pellet diet (Ashirwad Industries, Mohali) and clean drinking water ad libitum during the whole duration (56 days) in institutional CAF until euthanasia.

### 2.3. Plant Material and Formulation of the Extract

Citrus grandis (L.) Osbeck (grapefruit) fruit was collected from Saharanpur (Uttar Pradesh, India) and subsequently used for obtaining the peel. The plant material was validated by Dr. Sunita Garg, Emeritus scientist, Council of Scientific and Industrial Research - National Institute of Science Communication and Policy Research (CSIR-NISCAIR), New Delhi (India), and a specimen was submitted and preserved in this institute for future reference (Ref. voucher no. RHMD/2016/2998-25-1). The plant sample (peel of Citrus grandis) was shade dried and ground. The samples were examined for not containing any of the white flesh under the peel. The ground material (60 g) was extracted for 72 hours using aqueous ethanol (80%) in the Soxhlet apparatus. The extract was sieved (Whatman paper) and concentrated to aridity under low compression in a revolving evaporator at 45-55°C yielding 12.5% (*w*/*w*) peel extract. The extract yield was 18.5%. The extract was kept at -20°C until usage. Peel extract was suspended in 0.5% sodium CMC (doses 100, 200, and 400 mg/kg).

### 2.4. Total Phenolic Content

The Folin-Ciocalteu test was intended to measure phenolic content from the extract. In the first instance, 3.5 ml of distilled water (H_2_O) and 0.25 ml of Folin-Ciocalteu mixture were mixed with 0.25 ml of the extract diluted, and 20% Na_2_CO_3_ was added after 3 minutes. The test tubes were set at 40°C for 40 minutes before a double-beam spectrophotometer measured the absorbance at 685 nm. The overall phenolic content was measured in mg per g of extracts as an equivalent of gallic acid [18].

### 2.5. Total Flavonoid Content

In brief, 0.05 ml of crude extract was added with 1 ml of ethanol, 4 ml of distilled H_2_O, and 0.3 ml of 5% NaNO_2_ solution and then incubated. After 5 minutes, 0.3 ml of aluminium trichloride (AlCl_3_) reagent (10%) was added, and the assay blend was permitted to stand for 6 minutes. Subsequently, 2 ml of NaOH (1 M) was added. With distilled H_2_O, the final volume was made 10 ml. The assay blend was permitted to stand for 15 minutes. Optical density was assessed at 510 nm wavelength, and the outcome was articulated as mg rutin equivalent per g extract [19, 20].

### 2.6. Acute Oral Toxicity Study

To evaluate LD50 (median lethal dose), the Karber technique was used [21]. Different clusters of Wistar rats of either sex (*n* = 5, 200-220 g) were given a single C. grandis peel ethanolic extract (CGPE) dose (10, 100, 300, 2000, 5000, and 6000 mg/kg) by oral gavage. For acute toxicity study, Guideline 420 of the Organisation for Economic Cooperation and Development (OECD): Fixed-Dose Chemicals Test Procedure [22] was followed. Animals were independently monitored after dosing within the first 30 minutes at least once, regularly over the first 24 hours (with extra emphasis provided within the first 4 hours), and activity was observed for 48 hours. Observations involved modifications in skin and hair, eyes, and mucous membrane, as well as gastrointestinal, circulatory, autonomic, and central nervous (CNS) processes, and variations in somatomotor behavior and neurological behavior. Attention was guided to tremors, convulsions, salivation, vomiting, lethargy, fatigue, and coma monitoring.

### 2.7. Experimental Protocol

Thirty rats were randomly (single-blind method) separated into 2 collections: control (*n* = 6) and diabetic (*n* = 24). Control animals were given 0.5% sodium CMC vehicle and normal saline (5 ml/kg) only for 14 days daily. To induce diabetes, the animals fasted overnight, and a solitary intraperitoneal (i.p.) injection of freshly arranged alloxan (150 mg/kg in 0.9% w/v normal saline) was given on day 1 [23]. After 6 hours of administration of alloxan, glucose solution was provided orally in a feeding tube for 24 hours to resolve the early hypoglycemia arising from immediate major insulin release. After 3 days, 12 hours of fasting blood glucose (FBG) was measured by glucometer (ACCU-CHEK). The second drop of blood collected from the tail vein was used in ACCU-CHEK. Animals with glucose levels > 250 mg/dl were deemed diabetic. Diabetic animals were randomly distributed into following groups: diabetic control (DC), CGPE-L (low dose 100 mg/kg), CGPE-M (medium dose 200 mg/kg), CGPE-H (high dose 400 mg/kg), and Glib (5 mg/kg). C. grandis peel ethanolic extract (CGPE) or glibenclamide (Glib; 5 mg/kg) [24] was administered orally for 14 consecutive days to the diabetic rats. Diabetic control animals received an equivalent volume of 0.5% sodium CMC for 14 days daily. Blood glucose level was checked on days 1, 3, 7, and 14. Initial and final body weights were analyzed.

### 2.8. Biochemical Parameters

The blood sample was collected under light anesthesia (diethyl ether) by the sinocular puncture method in EDTA-containing tubes. The serum was detached by centrifugation of the blood sample at 2500 × g for 5 minutes at 4°C. Clear serum was used for the measurement of total cholesterol (TC), high-density lipoproteins (HDL), lactate dehydrogenase (LDH) rate, and creatine kinase (CK) rate. Lactate dehydrogenase (LDH) and creatine kinase MB (CK-MB) were determined as per the procedure given in kit booklets. Rats were sacrificed by cervical dislocation, and the heart was dissected out and rinsed in ice-cold isotonic saline. A 10% *w*/*v* cardiac tissue homogenate was made using freezing 50 mM potassium phosphate buffer and centrifuged at 10,000 × g for 15 minutes at 4°C to obtain clear supernatant. This supernatant was used to measure biochemical parameters. Thiobarbituric acid reactive substance (TBARS) was measured (nmoles/mg protein) by the method of Ohkawa et al. [25]. Ellman's [26] procedure was used for reduced glutathione (GSH) measurement (nmoles/mg protein). Superoxide dismutase (SOD) activity (IU per mg protein) was measured by following the method of Misra and Fridovich [27]. Catalase (CAT) activity (moles of H_2_O_2_ decayed per minute per mg protein) was assessed by the method given by Aebi [28]. ELISA kit was used for the evaluation of tumor necrosis factor-*α* (TNF-*α*). Total protein was computed by the technique of Lowry et al. [29]. For histological analysis, the cardiac tissues were preserved in a 10% formalin solution.

### 2.9. Histopathological Examinations

For histopathological evaluation, 4 *μ*m sections were developed by microtome and stained for 15 minutes with hematoxylin (H), followed by eosin (E) counterstain for 2 minutes. The slides were examined using a pathological microscope (Magnus) attached to a digital camera and software system.

### 2.10. Statistical Analysis

The statistical measurements used GraphPad Prism 5.01 (USA). The results were represented as mean ± standard mean error (SEM). A one-way ANOVA and Tukey's HSD tests were used to analyze the data. Time-course data were assessed using repeated measures two-way ANOVA and Bonferroni post hoc test. Statistical significance was considered at *p* < 0.05.

## 3. Results

### 3.1. Phenolic and Flavonoid Contents

The total phenolic content of CGPE was 46.23 ± 1.67 gallic acid equivalents/g (calibration curve *R*^2^ = 0.995) and the total flavonoid content 36 ± 1.56 rutin equivalents/g (*R*^2^ = 0.998).

### 3.2. Acute Oral Toxicity Investigation

The LD50 of CGPE was examined up to 6000 mg/kg dose. No symptoms of toxicity or death were evident at these doses. The observations revealed the nontoxic nature of the extract as all the animals were alive, healthy, and active during the observation period. CGPE had no influence on the change in behavior or general activity of the animals, and no death was observed at this dose. It can be inferred that the LD50 value of CGPE was more than 6000 mg/kg and is in the nontoxic range.

### 3.3. Effect of C. grandis Peel Ethanolic Extract on Body Weight and Blood Glucose Levels

The initial body weight and blood glucose level had no significant alteration. However, the mean body weight of the DC group on day 14 was considerably low in contrast to the control group. Oral administration of CGPE for 14 days daily attenuated the alloxan-induced decline in body weights of rats relative to DC rats (Figure 1(a)). Glib managed to attenuate the decrease in body weight in alloxan-treated rats when juxtaposed to rats that received alloxan and vehicle only. Injection of alloxan caused an increase in FBG on day 3 (>250 mg/dl). Rats treated with alloxan only showed a substantial rise in blood glucose levels on days 7 and 14 relative to the vehicle treated control rats. Treatment with CGPE or Glib significantly attenuated the alloxan-induced rise in blood glucose in rats when juxtaposed to rats that were given alloxan and vehicle only. Interestingly, we observed a dose-dependent decrease in blood glucose levels as shown in Figure 1(b).

### 3.4. Effect of C. grandis Peel Ethanolic Extract on Blood Biomarkers

DC group, administered with alloxan and vehicle only, showed a significant increase in serum TC levels, LDH activity, and CK activity and decline in HDL relative to the vehicle-treated control group (Figure 2). Oral administration of CGPE or Glib for 14 days in separate groups caused a noteworthy decrease in TC, LDH, and CK and a rise in HDL content in alloxan-treated rats when juxtaposed to rats that were given alloxan and vehicle only. The higher dose of CGPE (400 mg/kg) showed a conspicuous amelioration of blood lipid parameters and LDH and CK activities in comparison to the lower dose (100 mg/kg) in alloxan administered rats.

### 3.5. Effect of C. grandis Peel Ethanolic Extract on Oxidative Stress Biomarkers in Cardiac Tissue

The current findings depicted a substantial upsurge in lipid peroxidation (TBARS) and a diminution in cardiac antioxidants (GSH, SOD, and catalase) in retort to alloxan treatment when compared to the vehicle-treated controls (Figure 3). Treatment with CGPE or Glib attenuated alloxan-induced increase in TBARS and decline in antioxidants with respect to alloxan and vehicle alone treatments. Oral administration of CGPE-H dose caused a consistent decrease in TBARS and also enhanced the antioxidant levels steadily in the cardiac tissue in comparison to the lower dose, i.e., CGPE-L in alloxan-treated rats.

### 3.6. Effect of C. grandis Peel Ethanolic Extract on TNF-*α* in Cardiac Tissue

Analysis of ELISA results showed a significant rise in TNF-*α* (inflammatory biomarker) in cardiac tissue of alloxan-treated rats with respect to the vehicle-treated control rats. CGPE or Glib treatments for 14 days in alloxan treated rats significantly lowered the TNF-*α* levels relative to rats that received alloxan and vehicle only (Figure 4). The higher dose of CGPE (400 mg/kg) showed a conspicuous amelioration of inflammatory biomarkers in comparison to the lower dose (100 mg/kg) in alloxan administered rats.

### 3.7. Histopathology of Cardiac Tissue

Alloxan-induced diabetes caused significant pathogenic alterations in the heart of rats. DC group showed prominent changes in the plasma membrane, cell swelling, and chromatin condensation that highlighted the irreversible cell damage symptoms. Treatment with CGPE abrogated this alloxan-induced pathogenicity and showed a dose-dependent decline in cell deterioration. Glib also protected cell structure against alloxan-induced diabetes in rats (Figure 5).

## 4. Discussion

The research was aimed at determining the ameliorative effect of CGPE on DCM caused by alloxan. Alloxan is the most widely used entity for the induction of human insulin-dependent diabetes mellitus (IDDM) in laboratory diabetic animal models. When given intravenously, intraperitoneally, or subcutaneously, alloxan imposes its hyperglycemic actions. Alloxan has been reported to suppress the glucose-induced secretion of insulin by adaptive glucokinase deactivation and to cause IDDM. Due to a spurt in ROS (oxidative stress) and peroxides [30], alloxan has also been reported to induce a cytotoxic effect on pancreatic cells. Such free radical species cause oxidative and induced late inflammatory damage to the living systems [31]. In this investigation, a single-dose administration of alloxan (200 mg/kg, i.p.) caused persistent hyperglycemia that was attenuated by a 2-week CGPE or Glib treatment in rats.

In the diabetic control rats, the blood TC levels were increased, whereas HDL levels were reported to decrease. Earlier reports also indicate the level of TC in alloxan-induced diabetic rats to be increased [32]. However, treatment with CGPE or Glib (standard) was found to significantly decrease the TC and surge HDL. CGPE-H (400 mg/kg) showed the highest lipid-ameliorating activity among all CGPE treatment groups. The absence of flexibility between energy sources results in reduced heart efficiency and contractile dysfunction, which is a feature of cardiomyopathy in diabetics. The leakage of the cytoplasmic LDH caused by the damage to cell membrane integrity is reported as a reliable indicator of cell death and has been used to estimate the cytotoxicity [33]. It has been observed that an increase in the serum LDH levels indicates the nonspecific damaging response of any tissue [34]. The serum LDH levels were found to increase in the diabetic control rats. However, treatment with different doses of CGPE was found to attenuate the LDH levels significantly. Among all the different doses of C. grandis extract, CGPE-H was found to attenuate the LDH levels more significantly than other doses of it. An increase in serum levels of creatine kinase MB (CK-MB) has been used as a specific indicator of myocardial damage. This increase in CK-MB levels indicates cardiac muscular damage which results in leakage of enzymes from the heart and hence their elevated levels in the serum [10]. The CK-MB concentrations in the diabetic control rats were reported to be elevated. However, therapy with different doses of CGPE was found to greatly attenuate the CK levels. CGPE-H (400 mg/kg) has been found to ameliorate the CK-MB level more significantly among other CGPE dose groups. The present findings are in line with previous results that indicated amelioration of lipid profile, glucose metabolism, and attenuation of insulin resistance and cell death in different animal models [35]. Citrus fruits including C. grandis target diverse set of molecules such as PPARs, nuclear factor-*κ*B, platelet-derived growth factor (PDGF), transforming growth factor-1 (TGF-1), and genes, such as FAS, Progastricsin (PGC-1*α* and PGC-1*β*), and GLUT4 to prevent the progression of pathogenic mechanisms [35–37].

It has been confirmed that citrus phenolic compounds particularly flavonoids have significant antioxidant effects against radicals and anti-inflammatory properties. The citrus flavonoids are capable of trapping electrons and suppressing and/or scavenging the radicals. The citrus flavonoids create a tautomeric dislocation that prohibits certain oxygen-free radicals from propagating chain reactions [38, 39]. The heart disruption induced by hyperglycemia results in myocardial necrosis that triggers cardiac impairment, elevated lipid peroxidation, decreased myocardial lipid concentrations, and altered heart enzyme and antioxidant activity. As this research reveals that the amount of TBARS and TNF-*α* in diabetic control groups was observed to be increased. Nonetheless, treatment with 400 mg/kg of CGPE was found to significantly decrease the TBARS and TNF-*α* levels. Of all the doses of CGPE, the 400 mg/kg concentrations were observed to decrease lipid peroxidation and inflammation more than other doses and this disparity was significant. In diabetic control groups, the SOD activity, reduced glutathione level, and catalase rate were also observed to decrease. However, therapy with CGPE has been shown to dramatically improve these antioxidants.

Histopathological alterations arise in DCM characterized by necrosis; focal accumulation of chronic inflammatory cells comprised of lymphocytes, plasma cells, and macrophages; and edema [23]. In this research, the diabetic control group demonstrated the existence of granular cardiomyocyte degeneration, necrosis, perivascular edema, and extreme inflammatory cell infiltration. Treatment with CGPE or Glib attenuated necrosis and inflammatory cell infiltrations against DCM. CGPE was observed to reduce the inflammatory cells and recover the architecture of cardiomyocytes in the hearts of diabetic rats.

## 5. Conclusion

Present research indicates that chronic hyperglycemia is liable for heart muscle damage via the production of free radicals and inflammation. CGPE attenuated oxidative stress and inflammation in cardiac tissue and also lowered glucose levels and ameliorated lipid levels against alloxan-induced DCM in rats. The enhanced free radical generation acts as a chief position in the progression of DCM. Current insulin therapies that are used to control insulin resistance do not offer much protection against comorbidities, such as DCM. The use of crude phytochemicals as an adjuvant to current therapies continues to show benefits in various epidemiological and clinical studies. Hence, it may rule out some noxious side effects of synthetic drugs and widens the scope of a novel alternative therapy such as C. grandis peel extract in DCM.

## Figures and Tables

**Figure 1:** Effect of C. grandis peel ethanolic extract (CGPE) on (a) body weight and (b) blood glucose level. Repeated measures two-way ANOVA and Bonferroni post hoc test were used to analyze the data. Values are mean ± SEM (*n* = 6). ^##^*p* < 0.01 and ^###^*p* < 0.001 vs. control group; ^∗^*p* < 0.05 and ^∗∗∗^*p* < 0.001 vs. DC group; ^*ψψψ*^*p* < 0.001 vs. CGPE-L group; ^♦♦♦^*p* < 0.001 vs. CGPE-M group.

**Figure 2:** Effect of C. grandis peel ethanolic extract (CGPE) on blood biomarkers. (a) Total cholesterol level, (b) high-density lipoprotein (HDL), (c) lactate dehydrogenase (LDH) activity, and (d) creatine kinase MB activity. One-way ANOVA and Tukey's HSD post hoc test were used to analyze the data. Values are mean ± SEM (*n* = 6). ^###^*p* < 0.001 vs. control group; ^∗∗∗^*p* < 0.001 vs. DC group; ^*ψψψ*^*p* < 0.001 vs. CGPE-L group.

**Figure 3:** Effect of C. grandis peel ethanolic extract (CGPE) on oxidative stress biomarkers in cardiac tissue. (a) TBARS level, (b) glutathione (GSH) level, (c) superoxide dismutase (SOD) activity, and (d) catalase activity. One-way ANOVA and Tukey's HSD post hoc test were used to analyze the data. Values are mean ± SEM (*n* = 6). ^###^*p* < 0.001 vs. control group; ^∗∗∗^*p* < 0.001 vs. DC group; ^*ψψψ*^*p* < 0.001 vs. CGPE-L group.

**Figure 4:** Effect of C. grandis peel ethanolic extract (CGPE) on TNF-*α* in cardiac tissue. One-way ANOVA and Tukey's HSD post hoc test were used to analyze the data. Values are mean ± SEM (*n* = 6). ^###^*p* < 0.001 vs. control group; ^∗∗∗^*p* < 0.001 vs. DC group; ^*ψψψ*^*p* < 0.001 vs. CGPE-L group.

**Figure 5:** Histology of cardiac tissue. Cardiac photomicrograph (45x) showing usual anatomy with well-preserved cytoplasm. Diabetic control cardiac tissue shows clear penetration of inflammatory cells, the existence of lipid accumulation, swelling, ruptured, edema, and necrosis as indicated by arrows. Treatment with CGPE or Glib showed reduced, absence of lipid accumulation, inflammatory cells, and inflammation in cardiac tissue, the inflammatory cells decrease considerably, and partial cardiac tissue recovery is observed as shown by the arrows but shows some swollen and ruptured cells with lipid accumulation. There is a significant decrease in lipid accumulation, necrosis, and partial recovery of inflammatory cells, swollen, ruptured, and edema.

## Data Availability

The data is available from the corresponding author upon a suitable request.
